# Effect of Transdermal Fentanyl Patch Combined with Enhanced Recovery after Surgery on the Curative Effect and Analgesic Effect of Liver Cancer

This article has been retracted.

**DOI:** 10.1155/2022/9722458

**Published:** 2022-07-25

**Authors:** Hengmei Zhu, Hongmei Xiao, Guihua Lu, Shuheng Fang

**Affiliations:** ^1^Special Needs Diagnosis and Treatment Department, The Third Affiliated Hospital of Naval Military Medical University, Shanghai, 200438 Shanghai, China; ^2^Operating Room of Department of Anesthesiology, The Third Affiliated Hospital of Naval Medical University, Shanghai, 200438 Shanghai, China; ^3^Hematology Department, The First Affiliated Hospital of PLA Navy Medical University, Shanghai, 200438 Shanghai, China

## Abstract

Its goal was to see how a transdermal fentanyl patch combined with accelerated recovery after surgery (ERAS) affected the treatment efficacy and analgesic effect of liver cancer, as well as to help patients with liver cancer choose the right analgesic treatment and nursing mode. 150 patients with liver cancer were divided into group A (transdermal fentanyl patch), group B (ERAS), and group C (transdermal fentanyl patch combined with ERAS). Patients in the three groups were compared in terms of pain, survival, psychological status, adverse responses, postoperative recovery, and patient satisfaction. The results showed that under different treatment and nursing methods, the number of patients with mild cancer pain in the three groups was increased, especially the number of patients with mild cancer pain in group C (*P* < 0.05). Besides, the quality of life score of patients in each group was decreased. Patients who received the combination analgesia had a significantly higher quality of life than those who received simply a transdermal fentanyl patch or ERAS (*P* < 0.05). The scores of both the Hamilton anxiety scale (HAMA) and Hamilton depression rating scale (HAMD) of patients with the combined analgesia were decreased signally (*P* < 0.05). There were few patients with combined analgesia who had adverse reactions (*P* < 0.05). After surgery, the time of the first anal exhaust, first defecation, and first ambulation in group C were shorter than those in the other two groups (*P* < 0.05). To summarize, combining the two techniques aided in the recovery of gastrointestinal function as well as the physical recovery of patients following surgery. Furthermore, combining the two approaches produced a clear analgesic impact, which could improve patients' quality of life while also having a favorable clinical adoption effect.

## 1. Introduction

Liver cancer is very common in malignant tumors, whose main cause is chronic hepatitis B [1]. People have been paying greater attention to health examinations in recent years. Early detection and diagnosis of liver cancer can anticipate and identify the disease at an early stage, giving patients a variety of treatment options [2]. Pain is the most severe and excruciating clinical symptom for patients with liver cancer, affecting their physical and mental health, making daily life inconvenient, and affecting patients' regular daily lives, resulting in sadness. Cancer pain can make patients anxious and irritable, which makes it difficult to eat and sleep properly and brings serious problems for the patients [3, 4]. Besides, it makes the patient's treatment compliance worse, and they are unwilling to accept relevant treatment. As a result, tumor treatment efficacy is diminished, and the length of hospital stay is prolonged, putting a financial strain on the patient's family [5, 6]. Currently, both drug and nondrug therapies are the main treatment methods for cancer pain [7]. Drug therapy is majorly the use of analgesic drugs to relieve pain. The analgesic effect is obvious and quick, and the operation is convenient, with high patient acceptance. However, various analgesics have many side effects, including nausea, vomiting, constipation, and vertigo, which bring certain pain and cause great physical damage to patients [8]. Nondrug treatment includes surgical treatment, radiotherapy, and chemotherapy, all of which are difficult to operate on and result in severe injuries, with many complications, high cost, and adverse reactions [9].

Drug therapy is still the primary way to control cancer pain due to its convenient operation and high compliance of patients [10]. Fentanyl is an opioid receptor agonist, which can be absorbed through the skin, with a good effect of relieving pain [11]. Transdermal fentanyl patch can be absorbed directly through the skin. As a strong opioid, it is easy to operate on, and it can greatly relieve the pain of cancer patients, with stable effect and strong reliability [12]. However, in the treatment of cancer pain, transdermal fentanyl patches have several side effects, the most common of which are rash and pruritus [13]. The transdermal fentanyl patch offers a precise and stable analgesic effect, especially for moderate and severe cancer pain, and can help patients feel better after surgery with fewer side effects [14]. Enhanced recovery after surgery (ERAS), also known as fast track surgery (FTS), is a new concept, which is coordinating various disciplines to promote the rehabilitation of patients [15]. This nursing method entails reducing all unnecessary surgeries, reducing patient injury and stimulation, decreasing treatment pain and psychological stress, and improving patient comfort [16]. The main contents of ERAS include strengthening preoperative propaganda and education, shortening preoperative fasting and drinking time, timely analgesia for patients, early removal of the drainage tube, guidance for patients to get out of bed as soon as possible, and resuming oral feeding as soon as possible [17]. It can improve patients' comfort, reduce their treatment pain, and relieve bad emotions [18]. ERAS is a humanistic nursing model that focuses on the needs of patients and offers them targeted and comprehensive nursing care as well as psychological therapy. It is supported and recognized by patients in clinical practice, with a good adoption value.

Different treatment and nursing methods were used in 150 patients with liver cancer. The efficacy and analgesic effect of transdermal fentanyl patch alone, ERAS alone, and transdermal fentanyl patch combined ERAS on patients with liver cancer were compared. With different treatments and nursing, the analgesic effect, psychological state, postoperative recovery, and satisfaction of patients were compared among the three groups. Moreover, the efficacy of the three groups was analyzed, which was hoped to provide guidance and reference for pain relief and treatment of patients with liver cancer.

The rest of the paper is organized as Section 2 gives materials and methods, Section 3 gives us results, Section 4 provides discussion, and the conclusion is given in Section 5.

## 2. Materials and Methods

In this section, we will discuss research objects, methods, observation indexes, and statistical treatment in detail.

### 2.1. Research Objects

150 patients with liver cancer who were admitted to the hospital between January and December 2020 were chosen as research subjects, and they were divided into three groups on average. Patients in group A received only the transdermal fentanyl patch, patients in group B received only ERAS, and patients in group C received both the transdermal fentanyl patch and ERAS. This experiment was approved by the ethics committee of the First Affiliated Hospital of PLA Navy Medical University.

The inclusion criteria were as follows:

1. Patients with complete medical record
2. Patients who were able to communicate normally with the nurse
3. Patients without genetic diseases
4. Patients who signed the informed consent

The exclusion criteria were as follows:

1. Patients who had difficulty communicating normally
2. Patients with other malignancies
3. Patients who were unwilling to participate in the experiment

### 2.2. Methods

Group A was treated with the transdermal fentanyl patch. The specific methods were as follows. A transdermal fentanyl patch (Changzhou Siyao Pharm Co. Ltd., H20057054) was affixed to the patient's skin and applied immediately after opening to maintain its good efficacy. The patch was firmly set and did not fall off by pressing the area where it was glued with the palm. Each time, the dosage was 4.2 mg, and the duration was 0.5 minutes. Every three days, the patch had to be replaced, and the position had to be altered. The patch dose needs to be increased if the patient's pain relief wasn't noticeable.

Patients in group B received ERAS. The methods were as follows:

For preoperative nursing:

1. The fundamental information of the patients was examined, the patients were instructed to obtain standard hospital tests, imaging films were taken to grasp the tumor's relevant status, and a realistic surgical plan was made as part of the health evaluation
2. For health education, professional disease guidance was provided, and the occurrence principle, clinical manifestations, coping methods, common complications, and adverse reactions were explained to the patients. Besides, patients were informed how to avoid the occurrence of adverse reactions and how to deal with them after the occurrence. Food recommendations were based on needs, dietary contraindications were explained, and a diet conducive to disease remission was suggested
3. For preoperative drug preparation, patients were instructed to take 800 mL 5% glucose orally the night before surgery and the 250 mL glucose orally 2 h before surgery, and the antibiotics were injected half an hour before surgery to prevent postoperative infection
4. The relocation of intestinal flora might be avoided, as well as the occurrence of intestinal edema and intestinal paralysis, without the use of a preoperative enema and indwelling gastric tube for preoperative gastrointestinal management. Furthermore, pharyngeal discomfort caused by an indwelling gastric tube may be avoided, lung infection could be decreased, patient pain could be addressed, and patients' psychological and financial burdens might be reduced

For intraoperative nursing:

1. Short-acting anesthetics were utilized for patients to improve early recovery of consciousness following surgery and limit the effects of anesthetics on the nerve and endocrine function, according to the anesthesia selection
2. For accurate surgery, guided by imaging, surgical resection of the lesion could reduce the injury of the wound, preserve the liver function of the patient as much as possible, and promote the recovery of them
3. The patient's vital signs were monitored during the operation, the infusion volume was regulated for control, and patients received enough oxygen
4. For body temperature protection, during the surgery, it was necessary to keep the patient warm. The indoor temperature needed to be adjusted in time, and the operating room temperature needed to be maintained at 24-25 °C. The thermal insulation pad and thermal insulation blanket were used for the patient, and the thermal insulation measures were implemented, thus preventing the patient from low temperature during the surgery and reducing the occurrence of related complications. During the surgery, the patient's privacy needed to be safeguarded, and the body needed to be covered timely to maintain the dignity of the patient

For postoperative nursing:

1. The liver surgery incision was large, the patient's body harm was substantial, and the postoperative pain was noticeable, according to pain nursing. First, the severity of the patient's discomfort was determined, and effective analgesic measures were administered to relieve the patient's pain as soon as possible
2. For the nursing of the tube, the gastric tube and catheter were removed within 24 h after surgery so that the patient's gastrointestinal function could be restored as soon as possible to prevent the urinary tract infection
3. For diet guidance, after surgery, the patient was supplemented with nutrition to promote gastrointestinal peristalsis and accelerate the recovery of the patient's physique. If the patient did not have nausea or vomiting and was recovering well, the fluid diet could be augmented. The patient could be given warm water and clear liquids 6 hours after waking up under general anesthesia, with a gradual transition to semifluid food, soft food, and a normal diet
4. For postoperative activity guidance, patients were encouraged to get out of bed as early as possible after surgery, which was helpful to promote the metabolism, making the incision heal earlier, and preventing urinary retention and deep venous thrombosis. On a postoperative day, the patient could be assisted to turn over and be guided to clench fists and loosen fists.  Figure 1 showed the nursing process of ERAS

Patients in group C were treated with the transdermal fentanyl patch combined with ERAS.

### 2.3. Observation Indexes

The numeric rating scales (NRS) were used to measure cancer pain in patients for the classification of cancer pain. The highest possible score was 10. The more acute the pain, the higher the score. Mild was defined as 1-3 points, moderate as 4-6, and severe as 7-10.

For the quality of life scores, the functional living index-cancer (FLIC) was adopted. The higher the score was, the better the quality of life was.

For the anxiety and depression of patients, the Hamilton anxiety scale (HAMA) and Hamilton depression scale (HAMD) were adopted. The higher the score was, the heavier the degree was. When HAMA >14 points, it was anxiety. When HAMD >17 points, it was depression.

The main adverse reactions were constipation, vomiting, vertigo, and drowsiness.

The period of first anal exhaust, first defecation, and first ambulation were all measured for postoperative recovery.

The satisfaction evaluation form was created, and the patients who participated in the study were invited to fill it out to rate their satisfaction on a scale of 100. 80-100 points represented that patients were very satisfied, 60-80 represented that they were satisfied, and 0-60 represented that the patients were dissatisfied. Equation (1) showed how the patients' satisfaction was calculated. In Equation (1), *V* presented the number of patients who were very satisfied cases, *S* presented the number of patients who were satisfied, *D* presented the number of dissatisfied patients, and *Z* presented the total number of patients:

(1) $$\begin{array}{c} \text{Satisfaction}=\frac{\text{V}+\text{S}}{\text{Z}}\times 100\%. \end{array}$$

Figure 2 showed the observation indexes.

### 2.4. Statistical Treatment

PSS 20.0 was employed for data statistics and analysis. The *t*-test was used, and percentage (%) was how count data were expressed. The difference was statistically significant with *P* < 0.05.

## 3. Results

In this section, we will discuss the comparison of grading of cancer pain among three groups before and after treatment, comparison of quality of life scores among three groups before and after treatment, comparison of anxiety and depression among three groups before and after treatment, comparison of adverse reactions among three groups, comparison of postoperative recovery among three groups, and comparison of patients' satisfaction among three groups in detail.

### 3.1. Comparison of Grading of Cancer Pain among Three Groups before and after Treatment

Figure 3 showed the comparison of the grading of cancer pain in the three groups before and after treatment. Figures 3(a)–3(c) showed the number of patients with mild cancer pain, moderate cancer pain, and severe cancer pain. Before treatment, there was no statistical difference in the number of patients with mild, moderate, and severe cancer pain among the three groups (*P* > 0.05). In group A, there were 18 patients with mild cancer pain, 20 patients with moderate cancer pain, and 12 patients with severe cancer pain after therapy and nursing in various methods. There were 19 patients in group B who had mild cancer pain, 22 who had moderate cancer pain, and 9 who had severe cancer pain. There were 25 patients in group C with mild cancer pain, 18 with moderate cancer pain, and 7 with severe cancer pain. As a result, the number of patients with mild cancer pain increased in all groups following therapy, but the number of patients with moderate and severe cancer pain reduced. The increased number of patients with mild cancer pain in group C was more than that in group A and group B, and the number of patients with severe cancer pain was decreased notably (*P* < 0.05).

### 3.2. Comparison of Quality of Life Scores among Three Groups before and after Treatment

Figure 4 showed the comparison of quality of life scores among the three groups before and after treatment. There were no statistically significant changes in physical well-being, psychological well-being, cancer-related suffering, social well-being, or nausea scores between the three groups before treatment (*P* > 0.05). The above five scores of patients in each group reduced after varied therapies and care. Physical well-being was reduced to 23.52, psychological well-being was reduced to 17.62, cancer-related suffering was reduced to 4.72, social well-being was reduced to 3.87, and nausea score was reduced to 4.72 in group C. Group C's quality of life scores were significantly worse than those of groups A and B (*P* < 0.05).

### 3.3. Comparison of Anxiety and Depression among Three Groups before and after Treatment

In Figure 5, the HAMA scores were compared among the three groups before and after treatment. Before treatment, the differences were not statistical in HAMA scores among the three groups (*P* > 0.05). After treatment and nursing in different ways, the HAMA scores of group A, group B, and group C were decreased to 12.37, 10.78, and 6.54, respectively. The HAMA score in group C was decreased greatly (*P* < 0.05). The HAMD scores of the three groups before and after treatment are compared in Figure 6. Before treatment, the differences were not statistical in HAMD scores among the three groups (*P* > 0.05). After different methods of treatment and nursing, the HAMD scores of group A, group B, and group C were decreased to 13.69, 11.52, and 7.64, respectively. The decrease of HAMD score in group C was absolutely greater (*P* < 0.05).

### 3.4. Comparison of Adverse Reactions among Three Groups

Figure 7 showed the comparison of adverse reactions among the three groups. Figures 7(a)–7(d) showed the conditions of constipation, vomiting, vertigo, and drowsiness. In group A, there were 11 patients with constipation, 6 patients with vomiting, 8 patients with vertigo, and 3 patients with drowsiness. In group B, there were 10 patients with constipation, 5 with vomiting, 7 with vertigo, and 3 with drowsiness. In group C, 7 patients had constipation, 3 had vomiting, 3 had vertigo, and 1 had drowsiness. The number of adverse reactions in group C was evidently less than that of the other two groups (*P* < 0.05).

### 3.5. Comparison of Postoperative Recovery among Three Groups

Figures 8–10 showed the time of the first anal exhaust, time of the first defecation, and time of the first ambulation in the three groups after surgery. Compared with group A, the time in both group B and group C was observably shorter, and it was shortest in group C (*P* < 0.05).

### 3.6. Comparison of Patients' Satisfaction among Three Groups

Figure 11 showed the comparison of patients' satisfaction among the three groups. In group A, 15 patients were very satisfied, 26 were satisfied, and 9 were dissatisfied. In group B, 16 patients were very satisfied, 24 were satisfied, and 10 were dissatisfied. In group C, 19 patients were very satisfied, 26 were satisfied, and 5 were dissatisfied. Hence, patients who were very satisfied and satisfied in group C were manifestly more than those in the other two groups, with the highest satisfaction rate of 90% (*P* < 0.05).

## 4. Discussion

Liver cancer is common cancer, and its clinical symptoms mainly include fever, fatigue, and liver function damage [19–21]. With a high incidence of pain and severe cancer pain, the pain in the late stages of liver cancer is terrible and unbearable for patients. Treatment and nursing must include pain alleviation for patients [22]. The pain in liver cancer patients is mostly severe and persistent, so analgesic measures are necessary. Many liver cancer patients have pain as a result of their treatment methods and drugs, and patients experience evident pain symptoms following surgical resection of their liver cancer, which has a significant impact on their daily lives [23]. The main method for relieving the pain of patients is drug analgesia. Currently, the three-step analgesia therapy recommended by the World Health Organization (WHO) is generally adopted in medicine, and the selection of appropriate drugs based on the grading is recommended [24, 25]. Patients' pain can be effectively relieved by selecting appropriate medicine types and dosages based on the intensity of their discomfort. Furthermore, the bad effects are minor, the prevalence of adverse reactions is rare, and the patient harm is minimal. Opioids are analgesic drugs with good efficacy and high recognition. They can regulate afferent impulses, activate inhibitory pathways, and reduce the release of neurotransmitters [26]. As an opioid, fentanyl has a substantial analgesic effect [27]. ERAS is a new nursing mode with humanistic care, which is helpful to relieve patients' mental pressure, relieve their treatment pain, protect their dignity, and improve their comfort [28–30]. ERAS argues for the elimination of some unnecessary nursing procedures, such as the use of a stomach tube and a urinary tube, in order to prevent physical and psychological harm to patients while maintaining good patient recognition. Multimode combined analgesia is a new analgesic concept, which refers to the adoption of two or more than two methods for combined analgesia to achieve the ideal analgesic effect. It has a synergistic effect, which can improve the analgesic effect and reduce the incidence of complications [31, 32]. Drug treatment and nursing measures are very important to pain relief. Drug treatment can relieve the pain directly, whose effect is fast and substantial, and it has a good targeted effect on patients with acute unbearable pain. The nursing measure is a consistent and ongoing method of pain management that has a mild and long-term efficacy in reducing bodily and psychological pain. The patient's physical damage is small, and the patient's psychological acceptance is high. It plays a crucial role in the pain relief of patients with cancer. The combined analgesia is the combination of various analgesic methods, which relieves the patient's pain to the maximum extent. It has a good overall effect, with a noticeable analgesic effect, low adverse effects, high patient psychological acceptance, and high satisfaction. As a result, it has a high rate of clinical acceptance. Wan et al. (2021) [33] found that oxycodone combined with flurbiprofen and axitinib for analgesia in patients with colorectal cancer could effectively reduce pain intensity, especially visceral pain, and it helped reverse immunosuppression during radical colorectal cancer resection. Li et al. (2021) [34] pointed out that compared with the three-step analgesia alone, acupuncture combined with three-step analgesia could increase the reaction rate of pain relief in the treatment of cancer pain, reduce the side effects, reduce the rate of sudden pain, shorten the onset time of analgesia, and prolong the duration of the reaction.

The experiment assessed the analgesic effects, quality of life scores, anxiety and depression, adverse reactions, postoperative recovery, and patient satisfaction with the transdermal fentanyl patch alone, ERAS alone, and transdermal fentanyl patch paired with ERAS for liver cancer patients. The findings revealed that when different treatment and nursing methods were used, the number of cases of mild cancer pain increased in all three groups, while the number of cases of moderate and severe cancer pain decreased. Compared with the other two groups, the number of mild cancer pain in group C was signally higher, but that of severe cancer pain was reduced (*P* < 0.05). After treatment and nursing in different ways, the five scores of patients in each group were decreased. In group C, the decline of all the quality of life scores was remarkably greater compared with the other two groups (*P* < 0.05). It indicated that transdermal fentanyl patch combined with ERAS was conducive to the pain relief and improvement of life quality of patients. After different methods of treatment and nursing, the HAMA score and HAMD score of group C were decreased markedly (*P* < 0.05). The combined analgesia of the two modes could obviously relieve the anxiety and depression of patients. Compared with group A and group B, the number of adverse reactions in group C was evidently decreased (*P* < 0.05). It demonstrated that the combined analgesia of the two modes had fewer adverse reactions, with high safety. After surgery, the time of the first anal exhaust time, the first defecation, and the first ambulation in group B and group C were observably shorter compared with group A, and the time in group C was the shortest (*P* < 0.05). ERAS was more favourable to postoperative gastrointestinal function and physical recovery than the transdermal fentanyl patch, and the combination of the two treatments produced an optimal clinical impact. Furthermore, patients in group C were more satisfied than those in the other two groups, indicating that the transdermal fentanyl patch paired with ERAS was well-recognized by patients and had a high adoption rate.

## 5. Conclusion

The effects of different analgesic methods on pain relief and efficacy in patients with liver cancer were compared in this work. The results showed that transdermal fentanyl patch combined with ERAS had a good effect on pain relief, which could not only improve the quality of life of patients but also reduce the occurrence of adverse reactions. Moreover, it was beneficial to postoperative recovery, and it had high recognition from patients. In conclusion, it was a superior way to relieve pain, with great clinical adoption value.

## Figures and Tables

**Figure 1:** The nursing process of ERAS.

**Figure 2:** The observation indexes before and after treatment.

**Figure 3:** Comparison of the grading of cancer pain in the three groups before and after treatment. (a)–(c) The number of patients with mild cancer pain, moderate cancer pain, and severe cancer pain. Note: ∗ meant that the difference was statistically considerable before and after treatment, *P* < 0.05.

**Figure 4:** Comparison of quality of life scores among the three groups before and after treatment. (a)–(e) Physical well-being, psychological well-being, hardship caused by cancer, social well-being, and nausea scores. Note: ∗ meant that after treatment, compared with group A and group B, *P* < 0.05.

**Figure 5:** Comparison of the HAMA scores among the three groups before and after treatment. Note: ∗ meant that the difference was statistically considerable before and after treatment, *P* < 0.05.

**Figure 6:** Comparison of the HAMD scores among the three groups before and after treatment. Note: ∗ meant that the difference was statistically considerable before and after treatment, *P* < 0.05.

**Figure 7:** Comparison of adverse reactions among the three groups. (a)–(d) Constipation, vomiting, vertigo, and drowsiness). Note: ∗ compared with group A, *P* < 0.05.

**Figure 8:** Time of first anal exhaust after surgery in three groups. Note: ∗ compared with group A, *P* < 0.05.

**Figure 9:** Time of the first defecation after surgery in three groups. Note: ∗ compared with group A, *P* < 0.05.

**Figure 10:** Time of the first ambulation after surgery in the three groups. Note: ∗ compared with group A, *P* < 0.05.

**Figure 11:** Comparison of patients' satisfaction among the three groups.

## Data Availability

The experimental data used to support the findings of this study are available from the corresponding author upon request.
